# Phytochemistry and Biological Properties of *Salvia verbenaca* L.: A Comprehensive Review

**DOI:** 10.1155/2022/3787818

**Published:** 2022-05-24

**Authors:** Hanae Naceiri Mrabti, Naoual El Menyiy, Saoulajan Charfi, Mohammed Saber, Saad Bakrim, Reema A. Alyamani, Abdur Rauf, Ahmed M. H. Ali, Emad M. Abdallah, Naserddine El Omari, Abdelhakim Bouyahya, Hamza Assaggaf

**Affiliations:** ^1^Laboratory of Pharmacology and Toxicology, Bio Pharmaceutical and Toxicological Analysis Research Team, Faculty of Medicine and Pharmacy, Mohammed V University in Rabat, BP 6203 Rabat, Morocco; ^2^Laboratory of Pharmacology, National Agency of Medicinal and Aromatic Plants, Taounate, 34025, Morocco; ^3^Biology and Health Laboratory, Department of Biology, Faculty of Science, Abdelmalek-Essaadi University, Tetouan, Morocco; ^4^Laboratory of Nanotechnology, Materials and Environment, Department of Chemistry, Faculty of Science, Mohammed V University in Rabat, Morocco; ^5^Molecular Engineering, Valorization and Environment Team, Polydisciplinary Faculty of Taroudant, Ibn Zohr University, Agadir, Morocco; ^6^Faculty of Applied Medical Sciences, Clinical Nutrition Department, Umm Al-Qura University, Makkah 24381, Saudi Arabia; ^7^Department of Chemistry, University of Swabi, Khyber Pakhtunkhwa (KP), Pakistan; ^8^Department of Zoology and Entomology, Faculty of Science, Assiut University, Assiut, Egypt; ^9^Department of Science Laboratories, College of Science and Arts, Qassim University, Ar Rass, Saudi Arabia; ^10^Laboratory of Histology, Embryology, and Cytogenetic, Faculty of Medicine and Pharmacy, Mohammed V University in Rabat, Morocco; ^11^Laboratory of Human Pathologies Biology, Department of Biology, Faculty of Sciences, and Genomic Center of Human Pathologies, Faculty of Medicine and Pharmacy, Mohammed V University in Rabat, Morocco; ^12^Department of Laboratory Medicine, Faculty of Applied Medical Sciences, Umm Al-Qura University, Makkah 24381, Saudi Arabia

## Abstract

The family Lamiaceae contains several plants used in traditional medicine to fight against different diseases*. Salvia verbenaca* L. (*S. verbenaca*) is one of the Lamiaceae species distributed around the Mediterranean regions. This plant exhibits different bioactive properties, including antibacterial, anticancer, antioxidant, antileishmanial, antidiabetic, immunomodulatory, and wound healing. This review was conducted to revise previous studies on *S. verbenaca* addressing its botanical description, geographical distribution, and phytochemical, pharmacological, and toxicological properties. Moreover, the main pharmacological actions of *S. verbenaca* major compounds were well investigated. Literature reports have revealed that *S. verbenaca* possesses a pivotal role in medicinal applications. The findings of this work noted that *S. verbenaca* was found to be rich in chemical compound classes such as terpenoids, phenolics, fatty acids, sterols, and flavonoids. Numerous studies have found that *S. verbenaca* essential oils and extracts have a wide range of biological effects. These results support the potential pharmacological properties of *S. verbenaca* and its traditional uses. This analysis can constitute a scientific basis for further refined studies on its pure secondary metabolites. Therefore, the outcome of the present work may support the perspective of identifying new therapeutical applications with detailed pharmacological mechanisms of *S. verbenaca* to prevent the development of some diseases such as neurodegenerative disorders. However, toxicological investigations into *S. verbenaca* are needed to assess any potential toxicity before it can be further used in clinical studies.

## 1. Introduction

Since the beginning of time, medicinal plants have been and continue to be the primary source of medicine [1]. *Salvia verbenaca* L. (*S. verbenaca*) is a medicinal herb belonging to the family Lamiaceae, which is the most representative genus of *Salvia* [2, 3]. This plant is endemic to the Mediterranean region, including Morocco, Canaries Islands, Algeria, Tunisia, Libya, Egypt, and Cyprus, and has also spread to Europe and Asia [4]. In traditional medicines, *S. verbenaca* has been used to fight against numerous diseases; several ancient and current investigations revealed that *S. verbenaca* presents a chemical diversity in terms of chemical composition according to the chemical characteristics of the extracts from various parts. Indeed, *S. verbenaca* contains numerous secondary metabolites that belong to a wide variety of phytochemical classes [5]. *S. verbenaca* terpenoids have been revealed to have a large diversity due to several factors, including genetic, ecological, environmental, edaphic, and diverse plant parts [6]. An antibacterial potential against a wide range of gram-positive and gram-negative bacteria has been documented [7–11]. Consequently, the antibacterial efficacy of extracts and essential oils (EO) from *S. verbenaca* was remarkable against gram-positive bacteria compared to the gram-negative bacteria. Furthermore, *S. verbenaca* was found to have an antioxidant effect against free radical damage [12] and significantly reduce the level of intracellular reactive oxygen species (ROS) [13, 14]. According to previous studies, the anticancer properties of *S. verbenaca* extracts and essential oils have also been reported [15–19]. The antiparasitic properties of *S. verbenaca*, in particular, antileishmanial effects, have been investigated elsewhere [20].

Besides, *S. verbenaca* was reported to have an inhibitory effect of xanthine oxidase [21] and a healing effect on burns [22]. Furthermore, *S. verbenaca* revealed immunomodulatory effects [23]. Furthermore, the toxicological tests found that the ethanolic extract of *S. verbenaca* did not cause any toxic symptoms or death in rats [24].

The objective of the current article was to provide a general review of *S. verbenaca* such as botanical description, geographical distribution, phytochemistry, and pharmacological properties. Hopefully, this analysis could be a scientific basis for further refined studies on pure compounds from *S. verbenaca* that may lead to the identification of new therapeutical applications.

## 2. Research Methodology

All data about *S. verbenaca* (botanical description, taxonomy, destruction, phytochemical, and pharmacological properties) were collected using several databases like Web of Science, Google Scholar, Scopus, ScienceDirect, SpringerLink, Wiley Online, PubMed, and SciFinder and were reviewed in order to compile literature on *S. verbenaca*. The structures of the chemical profiles were identified in *S. verbenaca*, and the ChemDraw Pro 8.0 software was used to create the illustrations.

### 2.1. Botanical Description

*S. verbenaca* is a perennial herb that reaches between 10 and 50 cm (in height), hairy at the top, odorous, more or less glandular at the top. It grows in the dry lawns, the slopes, and at the edges of the paths. The slightly branched stems carry bunches of dark blue flowers in spring. Leaves are oblong, 2-3 cm broad, crenelated or incised-lobed, with the upper stalkless (Figure 1). The flowers are quite small, pale blue or whitish, in whorls usually close together, forming a fairly short cluster; the fruiting calyx with almost closed lips, bristling with spread hairs; the corolla is 10–15 mm, twice as long as the calyx, with wide lips, very uneven, the upper one compressed and curved in a false shape, and the style with little or prominent point [25].

### 2.2. Geographic Distribution

*S. verbenaca* has a very wide geographical distribution around the Mediterranean region, including Morocco, Algeria, Tunisia, Canaries, Egypt, Libya, Turkey, Cyprus, Transcaucasia, and Western and Southern Europe. It is also grown in South West Africa, North America, and Australia [5].

### 2.3. Ethnomedicinal Uses

The ethnobotanical investigations into *S. verbenaca* revealed its wide applications in folkloric medicine to treat numerous disorders as listed in Table 1. In Morocco, its application in folk medicinal systems includes the treatment of some digestive disorders such as abdominal colics [26–28]. The most commonly used part of the plant is the aerial part, which is prepared by infusion before being used to treat respiratory problems and genitourinary and skin diseases [27]. Dried leaves are also used for the treatment of wounds, burns, and abscesses [29]. Aerial parts are utilized in decoction or infusion to treat diabetes [30].

### 2.4. Phytochemistry

Like all medicinal plants belonging to the family Lamiaceae, *S. verbenaca* contains numerous secondary metabolites with different classes, such as flavonoids, terpenoids, alkaloids, and phenolic acids. Currently, several analytical investigations using different technical tools (GC, GC-SM, GC-MS, GC-FID, HPLC, 1D and 2D NMR, IR, UV, 1H NMR, and 13C NMR) have been applied to identify and isolate bioactive compounds from medicinal plants. Indeed, investigations into the chemical constituents of *S. verbenaca* revealed the presence of terpenoids, phenolics, fatty acids, flavonoids, and sterols (Table 2). As listed in Table 2, the chemical content of *S. verbenaca* was investigated in different areas with various medicinal applications by using different analytical tools. The results are different according to numerous factors, such as the study area, plant part used, and adopted methodology.

The terpenoids contained in the essential oils of *S. verbenaca* L. mostly consist of *α*-pinene, *β*-pinene, sabinene, 1,8-cineole, *β*-phellandrene, linalool, p-cymene, linalyl acetate, E-*β*-ocimene, (Z)-*β*-ocimene, tricyclene, camphor, 1,10-di-epi-cubenol, epi-13-manool, cis-muurola-3,5-diene, *δ*-selinene, *trans*-sabinene hydrate acetate, *β*-caryophyllene, viridiflorol, and germacrene D [31–33] (Table 1, Figure 2).

Belloum et al. [36] evaluated the volatile contents of the essential oil of *S. verbenaca* aerial parts using GC-MS and GC. In this sense, they recorded the presence of many terpenoids like germacrene D (20.5%), *β*-phellandrene (3.8%), *α*-copaene (10.4%), *β*-caryophyllene (3.8%), epi-*α*-cadinol (11.6%), and 1,10-di-epi-cubenol (20.9%). These compounds were the major terpenoids identified in *S. verbenaca* L. as reported elsewhere [31]. Moreover, in Spain, Taârit et al. [34] identified camphor (38.94%), 13-epi-manool (5.61%), and caryophyllene oxide (7.28%), from the essential oils of its seeds. A Greek study on *S. verbenaca* aerial parts has identified (E)-caryophyllene (16.1%) and *β*-phellandrene (30.3%) [34]. Moreover, Khemkham et al. [35] revealed *cis*-muurola-3,5 diene (14.6%) in the dried aerial parts of *S. verbenaca* as a major compound.

Al-Jaber et al. [25] compared the different parts of *S. verbenaca* volatile compounds collected from two locations in Jordan. Monoterpene hydrocarbons dominated the emission profile of stem, sepal, and leaf samples from the Mediterranean zone (68.0%, 33.7%, and 42.2%, respectively). Oxygenated monoterpenes controlled the production and emission of flowering components, including preflowering buds, fully grown flowers, and petals. Also, Taârit et al. [33] showed that the major compounds in EOs in *Salvia* aerial parts from the three Algerian regions were the monoterpene hydrocarbons and oxygenated sesquiterpenes. Additionally, the influence of collecting locations and phenophases on the production and chemical composition of *S. verbenaca* L. essential oils was examined by Farhat et al. [6]. In this study, it was reported that at the floral stage, monoterpene hydrocarbons (31.9%) prevail, whereas oxygenated sesquiterpenes (27.5%) predominate at the early fruiting stage. Sesquiterpene hydrocarbons were the most abundant chemical class at late fruiting (28.2%). Furthermore, Al-Jaber [32] reported that *S. verbenaca* EO was primarily composed of oxygenated monoterpenes (61.32%), with the monoterpene alcohol linalool serving as the sole monoterpene alcohol, whereas the essential oil obtained from the air-dried plant was primarily composed of sesquiterpene hydrocarbons (62.66%), with germacrene D serving as the major component (25.92%). Chemical heterogeneity of EOs was isolated from three distinct *S. verbenaca* tissues (leaves, twigs, and stem). In this regard, the EO of *S. verbenaca* from the fruits contains the highest concentrations of -caryophyllene (23.1%) and caryophyllene oxide (15.9%), while the EO from the stems contains the highest concentrations of camphor and viridiflorol and, and in comparison, the leaf oil contains the highest concentrations of epi-13-manool and manool [33].

Regarding phenolic acid compounds, several phenolic compounds were identified in the *S. verbenaca* methanolic extract, which was the phenolic acid with six compounds: p-hydroxybenzoic acid, vanillic acid, rosmarinic acid, p-coumaric acid, caffeic acid, phenolic diterpenes, and ferulic acid, with three compounds: carnosol, carnosic acid, and methyl carnosate [6] (Table 1, Figure 3). In Turkey, Tepe et al. [38] extracted rosmarinic acid from the dried methanolic extracts of this plant.

Moreover, Farhat et al. [6] have identified several flavonoids in methanol extract from aerial parts of Tunisian *S. verbenaca L* such as luteolin, apigenin, genkwanin, cirsiliol, naringenin, hesperidin, and naringin (Table 1, Figure 4).

Certain fatty acids were found in *S. verbenaca* (Table 1). Taârit et al. [33] identified approximately eight constituents (oleic acid, linoleic acid, arachidic acid, linolenic acid, palmitic acid, stearic acid, palmitoleic acid, and ethyl palmitate) (Figure 5). Russo et al. [19] isolated several interesting fatty acids from essential oils of *S. verbenaca* aerial parts, including (Z)-9-octadecenoic acid (oleic acid), hexadecanoic acid (palmitic acid), methyl hexadecanoate (methyl palmitate), and ethyl hexadecanoate (ethyl palmitate).

Additionally, Kabouche et al. [40] on the roots of *S. verbenaca* allowed the isolation of other secondary metabolites including five sterols (campesterol, stigmasterol, sitosterol, 6-hydroxysalvonolone, and microstegiol) and two diterpenes (6,7-dehydroroyleanone, cryptanol). Ahmed et al. [39] isolated two new diterpenes, namely, verbenacine and salvinine, from *S. verbenaca* aerial parts (Table 1, Figure 6).

### 2.5. Bioeffective Properties

Different parts of *S. verbenaca* exhibit the presence of several bioactive molecules of antibacterial, antileishmanial, antioxidant, and anticancer activities (Figure 7).

#### 2.5.1. Antibacterial Activity

The EOs and other organic extracts of *S. verbenaca* showed effective antibacterial effects against various gram-negative and gram-positive bacteria [7, 8, 10]. The inhibition zone diameter of *S. verbenaca* extracts and EOs and/or the minimum inhibitory concentration (MIC) are presented in (Table 3).

In Turkey, Sarac and Ugur [10] investigated the antibacterial potential of the ethanol extract from *S. verbenaca* aerial parts; they found that the extract showed a weak antibacterial activity, with IZD between 9 and 11 mm against the gram-positive bacteria *Staphylococcus epidermidis* (MU 30) (*Ф* = 9 mm), *Bacillus subtilis* (ATCC 6633) (*Ф* = 9 mm), *S. aureus* (MU 44) (*Ф* = 10 mm), *S. aureus* (MU 38) (*Ф* = 9 mm), and *S. aureus* (ATCC 25923) (*Ф* = 11 mm), and no activity was seen against *Streptococcus mutans* (CNCTC8/77) and *Micrococcus luteus* (NRRL B-4375) and nor gram-negative bacteria, *P. fluorescens* (MU87), *Escherichia coli* (ATCC25922), *Pseudomonas stutzeri* (MU70), *Pseudomonas aeruginosa* (ATCC27853), *Stenotrophomonas maltophilia* (MU64), *Chryseomonas luteola* (MU65), and *S. maltophilia* (MU99). Moreover, the ethanolic extract prepared from 12 *S. verbenaca* exhibited lower antimicrobial activity than the methanolic extracts, as found by Kostić et al. [9].

The investigation of the methanol extract from aerial parts of Tunisian *S. verbenaca* demonstrated that the extract had a high antibacterial potential (MIC = 500 *μ*g/mL) against six bacteria isolated from the mouths of patients [42]. However, a South African extract of *S. verbenaca* that was made with methanol and chloroform had strong antibacterial properties against *Klebsiella pneumoniae*, *Bacillus cereus*, *Escherichia coli*, and *Staphylococcus aureus* [11]. Moreover, Belkhiri et al. [21] compared the antibacterial potential of four fractions from the methanol extract of Algerian *S. verbenaca*: chloroform extract, crude extract, aqueous extract, and ethyl acetate extract. They have found that the antibacterial efficacy increases with the concentration of the extract. Al-Zereini [7] also found that the ethyl acetate extract prepared from the leaves of *S. verbenaca* from Jordan had dose-dependent antibacterial properties against *Bacillus brevis* (ATCC 9999) and *Bacillus subtilis* (ATCC 6633). On the other hand, the extract had no effect on *Klebsiella pneumoniae* (ATCC 13883), *Staphylococcus aureus* (ATCC 43300), and *Escherichia coli* (ATCC 25922). Canzoneri et al. [8] found that the EO of *S. verbenaca* aerial parts has potential antibacterial effects, and this activity is much higher against gram-positive bacteria than gram-negatives.

#### 2.5.2. Antioxidant Activity

The antioxidant potential of *S. verbenaca* extracts was investigated by several researchers [12, 21, 23, 38, 42–44], and Table 4 summarizes the majority of the investigations that were carried out on different parts of *S. verbenaca*, collected from different regions.

Kostić et al. [41] evaluated the antioxidant potential of different *S. verbenaca* extracts using the beta-carotene/linoleic acid system and DPPH assay. They found that the methanol extract had the highest activity in the DPPH method, while the ethanolic extract obtained by ultrasound extraction was the most active metabolite of beta-carotene/linoleic acid. The antioxidant activity of hydromethanolic extract prepared from stems and leaves of Moroccan species was carried out by Khlifi et al. [44]. The results showed that the extract had a significant antioxidant effect at 100 *μ*g/mL, with a strong inhibition of oxygen consumption compared to previous studies [38].

The antioxidant potential of Tunisian *S. verbenaca* extracts was also studied [42], and the results showed that methanolic extract from aerial parts had lower activity (IC_50_ = 86.9 *μ*g/mL) compared to the positive control, which was the trolox (IC_50_ = 23.12 *μ*g/mL) using the DPPH assay. In addition, it was reported that the antioxidant activity over 20 minutes using the ABTS assay increased with time, but was still four times lower than the activity of trolox. Additionally, Farhat et al. [6] studied the efficacy of the collection sites on the antioxidant capacity of methanolic extract prepared from postdistilled aerial parts of Tunisian species. They found that the site had a significant effect on the antioxidant potential by the DPPH, ABTS, and FRAP methods. Likewise, activity was shown to be substantially linked with total phenolic content.

The antioxidant activity of some extracts of *S. verbenaca* collected from Algeria was mostly studied using the DPPH assay. It was found that the crude extract prepared from aerial parts had good antioxidant activity that increased with increasing the extract concentration [14]. The scavenging activity was 95% at a concentration of 0.1 mg/mL. Also, the methanol extract of *S. verbenaca* aerial parts revealed a high reducing power in the FRAP test [43] using the DPPH assay. Additionally, it was cited that the methanol extract had a beneficial effect against free-radical damage and exhibited a 5-fold more inhibitory effect than the standard antioxidant trolox (IC_50_ = 72.63 *μ*M) [12]. They also observed that the radical scavenging activity had no significant correlation with the phenolic content and a low correlation with the flavonoid content. Belkhiri et al. [21] investigated the antioxidant potential of some fractions of the methanol extracts using the DPPH method, metal chelating activity, and reducing power assay, and all extracts showed potent antioxidant activity [13]. The cupric ion reducing capacity (CUPRAC) and Fe^3+^ reducing capacity (phenanthroline assay) of the extracts were investigated, and the findings exhibited that both extracts had high antioxidant capacity, with methanolic extract exhibiting the highest activity [14].

#### 2.5.3. Anticancer Activity

The different organic essential oils and extracts of *S. verbenaca* have been studied for anticancer properties. Numerous laboratory investigations using cell culture have shown that *S. verbenaca* extracts and essential oils have antiproliferative properties (Table 5) against a variety of cancer cell lines [15–19, 23, 45].

The ethyl acetate extract of *S. verbenaca* leaves produced after maceration was examined using the MDA cell lines MB-231 (human breast adenocarcinoma, ATCC HTB-26). The findings indicated that all extracts produced cytotoxicity in MDA MB-231 breast cancer cells [7]. However, it was proved that *S. verbenaca* leaf extracts possessed cytotoxic effect against HEp-2 (human larynx cancer cells) and Vero (monkey kidney cells) [18]. In another investigation, methanolic extracts of *S. verbenaca*'s aerial component prepared by maceration were evaluated in vitro against four human cancer cell lines, including HCA, HepG2, MCF-7, and HPC. The findings indicate that LC_50_ levels higher than 75 *μ*g/mL were deemed inactive [15]. Additionally, MTT assays were used to determine the cytotoxic activity of several extracts (methanol, hexane, ethyl acetate, n-butanol, and chloroform extracts) obtained from the aerial portion of *S. verbenaca* [16]. Methanol and chloroform extracts of *S. verbenaca* aerial parts were evaluated against colon adenocarcinoma (HT-29), human cancer cell lines (breast adenocarcinoma (MCF-7), human kidney epithelial cell line and glioblastoma (SF-268)) [17]. *S. verbenaca* exhibited more favorable action against MCF-7, with an IC_50_ value of 31.50 13.70 *μ*g/mL, but was inactive versus SF-268 and/or HT-29 cell lines [17].

A cell viability study was performed to avoid any cytotoxic concentration of *S. verbenaca* root extract on THP-1 cells. The MTT assay revealed that the most cytotoxic concentration of the extract was 1000 *μ*g/mL, which caused 70% of cell death and 30% of cell viability [23]. The essential oils of *S. verbena* were investigated for their ability to suppress the proliferation of human tumor cells using the human M14 melanoma cell line and shown significant efficacy [19]. The antiproliferative effect of *S. verbenaca* essential oil may be attributed to active sesquiterpenes in combination with other natural chemicals found in the essential oil components. Indeed, carvacrol and thymol exhibited outstanding anticancer properties through a variety of mechanisms [19].

#### 2.5.4. Antiparasitic Activity

Et-Touys et al. [20] investigated the antileishmanial effects of organic extracts (methanol, n-hexane, and dichloromethane extract) from *S. verbenaca*, and it was reported that the *in vitro* antileishmanial effect which was evaluated on the culture of three Leishmania species such as *Leishmania infantum*, *Leishmania tropica*, and *Leishmania major* was good (Table 6).

Belkhiri et al. [21] additionally observed that *S. verbenaca* has antihemolytic properties. In vitro antihemolytic activity of *S. verbenaca* extract was determined by inducing oxidative erythrocyte hemolysis. The results indicated that ethyl acetate extract was the most effective in inhibiting hemolysis, followed by crude extract, chloroform extract, and aqueous extract. Additionally, ethyl acetate extract inhibited hemolysis more effectively than vitamin C.

#### 2.5.5. Insecticidal Activity

In most cases, the application of synthetic pesticides is the primary approach for controlling insect pests, which produces excellent effects in a short period of time. Meanwhile, their irrational usage has resulted in global issues such as pollution, nontarget toxicity, biodiversity loss, and the development of pest resistance [46–48]. This need arose from a desire to provide alternatives to synthetic insecticides, which can have negative environmental consequences [49–52]. The insecticidal capabilities of *S. verbenaca* extracts and essential oils have been documented to have potential impact against several pests in previous studies [53]. Insecticidal action has been shown in several experiments using some *Salvia* species [54].

Essential oils from *Salvia* species revealed 100% repellency activity against adults of *Aedes albopictus* [55]. The oil of *S. verbenaca* drastically shortened the lifespan of *cowpea weevil* and prevented females from laying eggs [56]. Several crude extracts and essential oils from *Salvia* species were tested for pesticide activity against the test pest larvae [57–59]. Insectistatic and insecticidal properties of chloroform extracts from the aerial portions of four Salvia species were examined [60]. *S. verbenaca* extracts are very effective against *Culex quinquefasciatus* mosquitos [61]. Caryophyllene oxide was the major component in the essential oil of *S. verbenaca* with 7.28 [62]. The insecticidal activity and fumigant toxicity of caryophyllene oxide were tested against two insect pests, and it was shown to be effective [63].

### 2.6. Other Biological Effects

Different extracts from *S. verbenaca* have also exhibited other biological activities such as antihemolytic, immunomodulatory, and enzyme inhibitory effects (Table 7).

#### 2.6.1. Xanthine Oxidase Inhibitory Effect

Xanthine oxidase, abbreviated as XO, is an oxidoreductase that catalyzes the conversion of hypoxanthine to xanthine and xanthine to uric acid. Xanthine oxidase is generally present in the liver and in an inactive form in the blood in humans. A blood test for XO may identify liver impairment because xanthine oxidase is released into the blood in situations of severe liver injury [21].

#### 2.6.2. Burn Recovery Activities

Guaouguaou et al. [24] evaluated the impact of three *S. verbenaca* extracts on the healing of burns in rats using hexane, ethyl acetate, and n-butanol. The results indicated that various *Salvia verbenaca* plant extracts were more effective than silver sulfadiazine (SSD) and that it is the most widely used topical treatment for injury, with healed areas of 29.17% (base), 44.34% (hexane), 47.55% (ethyl acetate), 49.16% (n-butanol), and 41.09% SSD.

#### 2.6.3. In Vitro Antidiabetic Activity

Several earlier studies have shown *S. verbenaca*'s antidiabetic activity *in vitro* [13]. Additional studies are shown in Section 2.8 and Figure 8.

#### 2.6.4. Immunomodulatory Effects

Previous studies investigated the immunomodulatory effects of *S. verbenaca* aerial parts [14]. The carbon clearance rate test was used to determine the immunostimulant potential of this plant on phagocytic activity. The phagocytic index was much higher in rats who were given *S. verbenaca* at a dose of 200 mg/kg than in rats who were not given the herb.

### 2.7. Toxicological Investigations of *S. verbenaca*

The toxicological investigations of *S. verbenaca* have not been well studied. However, some studies carried out recently have confirmed the safety of these plant extracts (Table 8). Indeed, a report by Guaouguaou et al. [64] focused on the acute and subchronic effects of *S. verbenaca* toxicity in mice and rats through oral and topical administration. The findings of the acute toxicity of the fractions derived from *S. verbenaca* (n-butanol, hexane, and ethyl acetate) demonstrated that the LD_50_ of this plant after oral administration at 2000 mg kg^−1^ is not deadly [64]. In order to complete the toxicity profile of this plant, more research should be done to find out how toxic it is over a long period of time.

### 2.8. Pharmacological Properties of *S. verbenaca* Main Volatile Compounds

Several studies examined the major volatile chemicals found in *S. verbenaca*, including carvacrol, thymol, and linalool. Studies showed that carvacrol has hypoglycemic properties through intrinsic mechanisms such as blood glucose and insulin level lowering [65]. Additionally, carvacrol resulted in a drop in glucose levels. Additionally, these substances were shown to enhance the activity of glucokinase and glucose-6-phosphate dehydrogenase in the liver [66]. Carvacrol inhibits the enzymes *α*-amylase and alpha-glucosidase *in vitro* [67] and beta-galactosidase *in vitro* [68]. Thymol was also able to normalize blood sugar, plasma insulin, HbA_1c_, and the insulin resistance index in patients with hyperglycemia [69]. The levels of expression of genes involved in the production of insulin have been studied and reported in STZ-induced diabetic mice [70, 71], and a rise in *Mafa* and *Pdx1* gene expression has been reported. Limonene is another major constituent of *S. verbenaca* that has been shown to improve glucose homeostasis. Indeed, this substance boosts hepatic glycogen and plasma glucose levels [72] (Figure 8).

The antidiabetic effect has been also revealed by linalool (another main compound of *S. verbenaca*) [73, 74]. Indeed, linalool lowered blood glucose, hemoglobin A1c, fructosamine, interleukin-6, and tumor necrosis factor-*α* (TNF-*α*), while it increased insulin levels [74].

The major phytochemical compounds of *S. verbenaca* exhibited remarkable antibacterial effects [75–77]. Rhayour et al. [70] investigated the impact of thymol on gram-positive and gram-negative microorganisms, including *Bacillus subtilis* and *Escherichia coli* [75–78]. Antibacterial activity is demonstrated by modifying cell shape, damaging cell walls and membranes, and limiting the development of some types of bacteria, including *P. aeruginosa* [79]. In addition, limonene was found to be antibacterial because it targeted microorganisms' cytoplasmic membranes, weakened membrane integrity, blocked respiratory enzymes, and lost the proton motive force (Figure 9).

The anticancer properties of the major components in *S. verbenaca* (carvacrol, limonene, and thymol) have also been reported recently [80–82]. Thymol has been shown to have anticancer properties via a variety of mechanisms, including inducing severe DNA damage, including the production of reactive oxygen species (ROS) and subsequent increase in oxidative stress and/or mitochondrial dysfunction, or via the nuclear factor of activated T cell (NFAT-2) route [81]. Additionally, carvacrol increased apoptosis in cells, perhaps via activating mitochondrial apoptotic and signaling pathways [83].

## 3. Conclusions and Perspectives

*S. verbenaca*, a medicinal plant used in traditional medicine to cure a variety of ailments, was found to be abundant in bioactive chemicals such as flavonoids, terpenoids, and phenolic acids. Numerous pharmacological studies have demonstrated that *S. verbenaca* extracts and essential oils have extraordinarily beneficial effects on a variety of diseases, including those caused by microbes and those caused by dysregulation of homeostasis. Indeed, this plant demonstrated antibacterial, antidiabetic, anticancer, and immunomodulatory properties via a variety of mechanisms. However, further research should be conducted to find other pharmacodynamic targets. Additionally, pharmacokinetic studies should be conducted to ascertain the absorption, metabolism, and elimination of *S. verbenaca* bioactive components. Additionally, toxicological studies should be conducted to validate the safety of *S. verbenaca* extracts at various doses and delivery methods.

## Figures and Tables

**Figure 1:** *Salvia verbenaca* L.: (a) whole plant; (b) aerial part; (c) flowers.

**Figure 2:** Terpenoid structures identified from *S. verbenaca* EO.

**Figure 3:** Phenolic acids and phenolic diterpenes isolated from *S. verbenaca.*

**Figure 4:** Flavonoids of *S. verbenaca* extracts.

**Figure 5:** Some fatty acids isolated from *S. verbenaca* extracts.

**Figure 6:** Structure of compounds isolated from *S. verbenaca.*

**Figure 7:** Pharmacological properties of *S. verbenaca*.

**Figure 8:** Antidiabetic mechanism insights of *S. verbenaca* main compounds.

**Figure 9:** Suggested antibacterial mechanisms of *S. verbenaca* compounds.

**Table 1:** Some medicinal applications of *S. verbenaca.*

Part used	Preparation	Traditional application	Ref.
Aerial part	Decoction, infusion	Diabetes	[30]
Leaf	Decoction, powder	Abdominal colics, cold, fever, healing	[26]
Leaf	Powder	Wound treatment	[29]
Leaf	Decoction, infusion	Genitourinary, skin, digestive, and respiratory problems	[27]
Aerial part	No information	Digestive problems	[28]
Leaf, whole plant	Powder	Healing of burns, wounds, and abscesses	[29]

NI: no information.

**Table 2:** Chemical composition of various parts of *S. verbenaca.*

Part used	Country	Harvest site	Harvest season	Extracts/essential oils	Chemical composition	Analysis	References
Aerial parts (dry)	Tunisia	Rass Zebib (subhumid)	Flowering period	EO	1,8-Cineole (9.7%), p-cymene (8.4%), *α*-pinene (5.4%), *γ*-terpinene (3.1%), beta-caryophyllene (5.3%), viridiflorol (7.3%), epi-13-manool (4.7%), thymol (3.7%), limonene (2.8%), camphor (2.7%)	GC and GC-MS	[6]
Aerial parts (dry)	Tunisia	Bir Mroua (subhumid)	Flowering period	EO	*β*-Caryophyllene (15.3%), germacrene D (7.1%), epi-13-manool (6.2%), *α*-copaene (6.1%), *α*-humulene (4.3%), *α*-cadinol (3.9%), viridiflorol (3.4%), p-cymene (3.3%), *δ*-cadinene (3.1%), p-cymen-8-ol (2.6%)	GC and GC-MS	[31–33]
Aerial parts (dry)	Tunisia	Beja (higher semiarid)	Flowering period	EO	*β*-Caryophyllene (15.3%), *α*-humulene (3.0%), viridiflorol (11.6%), 1,8-cineole (3.3%), germacrene D (3.3%), (Z)-*β*-ocimene (4.0%), T-cadinol (1.9%), p-cymene (2.8%), thymol (2.7%), epi-13-manool (2.5%)	GC and GC-MS	[6, 31]
Aerial parts (dry)	Tunisia	Tunis (higher semiarid)	Flowering period	EO	Viridiflorol (17.7%), 1,8-cineole (8.5%), *α*-pinene (4.6%), p-cymene (5.2%), *β*-caryophyllene (5.5%), thymol (4.4%), epi-13-manool (4.0%), *α*-humulene (2.4%), *α*-thujone (3.6%), *γ*-terpinene (2.4%)	GC and GC-MS	[31, 33, 34]
Aerial parts (dry)	Tunisia	Touiref (moderate semiarid)	Flowering period	EO	*α*-Pinene (15.9%), camphor (4.7%), 1,8-cineole (12.8%), viridiflorol (10.0%), (Z)-*β*-ocimene (5.4%), camphene (2.6%), *β*-caryophyllene (5.3%), thymol (4.2%), p-cymene (4.2%), *α*-thujone (3.4%)	GC and GC-MS	[31, 33, 35]
Aerial parts (dry)	Tunisia	Bou Arada (moderate semiarid)	Flowering period	EO	1,8-Cineole (9.4%), p-cymene (8.7%), viridiflorol (8.3%), *α*-pinene (4.9%), thymol (2.7%), *β*-caryophyllene (4.9%), *α*-humulene (3.5%), *γ*-terpinene (3.0%), *α*-thujone (3.0%), epi-13-manool (3.6%)	GC and GC-MS	[31–33]
Aerial parts (dry)	Tunisia	Sers (lower semiarid)	Flowering period	EO	*α*-Pinene (14.7%), viridiflorol (10.8%), *β*-caryophyllene (4.6%), (Z)-*β*-ocimene (4.5%), epi-13-manool (2.8%), thymol (4.4%), p-cymene (4.1%), camphor (3.5%), *α*-thujone (2.9%), 1,8-cineole (10.9%)	GC and GC-MS	[31–33]
Aerial parts (dry)	Tunisia	Enfidha (lower semiarid)	Flowering period	EO	Viridiflorol (10.5%), camphor (2.9%), epi-13-manool (10.5%), 1,8-cineole (8.7%), p-cymene (8.3%), *α*-terpineol (3.0%), *α*-pinene (4.5%), thymol (4.2%), *γ*-terpinene (3.2%), bornyl acetate (3.2%)	GC and GC-MS	[31–33]
Aerial parts (dry)	Tunisia	Chott Meriem (higher arid)	Flowering period	EO	p-Cymene (14.2), *α*-pinene (9.6), *γ*-terpinene (5.1), camphene (3.9), viridiflorol (5.1), limonene (3.4), epi-13-manool (3.2), thymol (2.5), 1,8-cineole (12.8)	GC and GC-MS	[31–33]
Aerial parts (dry)	Tunisia	Hencha (higher arid)	Flowering period	EO	Viridiflorol (10.0%), bicyclogermacrene (2.3%), germacrene D (5.6%), 1,8-cineole (4.9), epi-13-manool (4.7%), *α*-thujone (3.2%), *β*-pinene (3.0%), camphor (2.9%), *α*-humulene (2.5%), *β*-caryophyllene (7.2%)	GC and GC-MS	[31–33]
Aerial parts (dry)	Spain	Murcia	Flowering stage	EO	p-Cymene (11.4%), 1,8-cineole (7.7%), viridiflorol (7.0%), camphene (2.7%), *β*-caryophyllene (4.5%), *β*-pinene (2.7%), *γ*-terpinene (4.0%), epi-13-manool (3.9%), camphor (3.7%), *α*-pinene (8.1%)	GC and GC-MS	[6]
Aerial parts (dry)	Spain	Murcia	Early fruiting stage	EO	Caryophyllene oxide (12.4%), bornyl acetate (3.2%), viridiflorol (9.1%), *β*-caryophyllene (5.6%), p-cymene (5.6%), *α*-pinene (4.0%), epi-13-manool (2.3%), thymol (2.0%), *β*-ionone (2.0%), 1,8-cineole (6.3%)	GC and GC-MS	[6]
Aerial parts (dry)	Spain	Murcia	Late fruiting stage	EO	*β*-Caryophyllene (14.2%), *α*-thujone (8.2%), 8-cineole (4.7%), epi-13-manool (7.1%), bornyl acetate (3.5%), *α*-humulene (6.7%), 1 *α*-pinene (4.3%), caryophyllene oxide (3.0%), *β*-pinene (2.8%), viridiflorol (13.5%)	GC and GC-MS	[6]
Aerial parts	Algeria	Bechar	April 2011	EO	Epi-*α*-cadinol (11.6%), *β*-caryophyllene (11.33%), bicyclogermacrene (10.9%), *γ*-cadinene (7.9%), *cis*-muurola-4(14),5-diene (7.8%), muurola-3,5-diene (5.2%), spathulenol (3.0%), *cis*-calamenene (2.0), *α*-humulene (1.9), 1,10-di-epi-cubenol (20.9%)	GC and GC-MS	[31]
Aerial parts (fresh)	Jordan	Shafa-Badran-Amman	Flowering period (April to May 2011)	EO	Linalool (61.32%), *β*-elemene (1.50%), (Z)*-β*-ocimene (4.03%), *β*-eudesmol (3.66%), spathulenol (3.40%), *E*-*β*-ocimene (2.63%), *β*-caryophyllene (2.98%), *α*-copaene (2.50%), *γ*-cadinene (1.55%), bicyclogermacrene (5.94%)	GC-MS and GC-FID	[32]
Aerial parts (dry)	Jordan	Shafa-Badran-Amman	Flowering period (April to May 2011)	EO	Linalool (30.72%), bicyclogermacrene (14.70%), *β*-caryophyllene (7.42%), germacrene D (25.92%), *α*-copaene (5.13%), isopentyl isovalerate (0.97%), *δ*-cadinene (2.05%), (Z)*-β*-ocimene (1.18%), spathulenol (1.58%), *α*-gurjunene (1.07%)	GC and GC-MS	[32]
Stem	Jordan	Mediterranean	Full maturation period	EO	*Z*-*β*-Ocimene (32.6%), *trans*-sabinene hydrate acetate (14.5%), *α*-gurjunene (6.0%), *β*-bourbonene (1.5%), *E*-*β*-ocimene (7.8%), sabinene (2.9%), *α*-phellandrene (3.1%), germacrene D (1.6%), *α*-pinene (9.3%), *β*-pinene (8.1%)	GC-MS and GC-FID	[32]
	Jordan	Irano-Turanian	Full maturation period	EO	*trans*-Sabinene hydrate acetate (38.1%), *E*-caryophyllene (9.1%), *δ*-selinene (5.2%), *β*-gurjunene (2.5%), sabinene (4.8%), *δα*-copaene (4.1%), *γ*-gurjunene (2.9%), cadinene (4.3%), *β*-selinene (2.2%), germacrene D (13.3%)	GC and GC-MS	[32]
Leaves	Jordan	Mediterranean	Full maturation period	EO	*trans*-Sabinene hydrate acetate (30.2%), *β*-bourbonene (7.7%), E-*β*-ocimene (4.3%), *α*-pinene (3.0%), *α*-gurjunene (13.8%), *β*-selinene (2.8%), *δ*-cadinene (2.5%), *β*-pinene (2.4%), myrcene (2.0%), Z-*β*-ocimene (17.1%)	GC and GC-MS	[32]
Leaves	Jordan	Irano-Turanian	Full maturation period	EO	*δ*-Selinene (21.5%), *E*-caryophyllene (11.4%), terpinolene (4.3%), *α*-copaene (9.6%), sabinene (9.0%), *Z*-*β*-ocimene (4.8%), *β*-cubebene (4.4%), *δ*-cadinene (2.7%), *cis*-*β*-guaiene (2.0%), germacrene D (19.8%)	GC and GC-MS	[32]
Preflower	Jordan	Mediterranean	Full maturation period	EO	*trans*-Sabinene hydrate acetate (56.5%), *α*-pinene (6.5%), myrcene (1.5%), *E*-*β*-ocimene (4.3%), *α*-gurjunene (3.2%), *β*-pinene (5.3%), sabinene (1.2%), *trans*-*β*-guaiene (1.0%), limonene (0.7%), *Z*-*β*-ocimene (13.5%)	GC and GC-MS	[32]
Preflower	Jordan	Irano-Turanian	Full maturation period	EO	Sabinene (42.7%), *α*-thujene (7.2%), *γ*-terpinene (6.1%), *E*-*β*-ocimene (1.9%), *α*-terpinene (3.6%), *β*-pinene (3.2%), *β*-phellandrene (6.8%), terpinolene (1.6%), limonene (1.0%), *trans*-sabinene hydrate (20.4%)	GC and GC-MS	[32]
Flower	Jordan	Mediterranean	Full maturation period	EO	*trans*-Sabinene hydrate acetate (58.6%), *E*-*β*-ocimene (5.3%), *α*-pinene (5.2%), sabinene (1.1%), *β*-pinene (4.9%), *α*-phellandrene (1.4%), *α*-gurjunene (1.0%), camphene (0.4%), isobornyl acetate (0.4%), *Z*-*β*-ocimene (18.8%)	GC and GC-MS	[32]
	Jordan	Irano-Turanian	Full maturation period	EO	Sabinene (37.5%), *Z*-*β*-ocimene (9.9%), *α*-thujene (4.6%), myrcene (4.2%), *β*-pinene (3.9%), *E*-*β*-ocimene (8.9%), *γ*-terpinene (3.0%), *E*-caryophyllene (1.9%), *α*-terpinene (1.4%), *trans*-sabinene hydrate (20.0%)	GC and GC-MS	[32]
Petal	Jordan	Mediterranean	Full maturation period	EO	*trans*-Sabinene hydrate acetate (87.0%), *E*-*β*-ocimene (1.5%), germacrene D (1.0%), *α*-phellandrene (0.5%), *β*-pinene (0.3%), *α*-gurjunene (1.7%), n-nonane (0.2%), myrcene (0.2%), *β*-selinene (0.2%), *Z*-*β*-ocimene (7.1%)	GC and GC-MS	[32]
Petal	Jordan	Irano-Turanian	Full maturation period	EO	*trans*-Sabinene hydrate (18.8%), *E*-*β*-ocimene (9.9%), *γ*-terpinene (2.9%), germacrene D (9.6%), *β*-copaene (4.1%), *α*-copaene (3.2%), *E*-caryophyllene (13.9%), *β*-selinene (2.9%), *γ*-gurjunene (2.8%), *Z*-*β*-ocimene (9.6%)	GC and GC-MS	[32]
Sepal	Jordan	Mediterranean	Full maturation period	EO	*trans*-Sabinene hydrate acetate (36.6%), *β*-pinene (14.0%), 8-cineole (3.9%), *Z*-*β*-ocimene (4.5%), 1 *δ*-elemene (2.8%), *β*-cedrene (8.7%), sabinene (2.7%), camphene (1.9%), *β*-cubebene (1.9%), *α*-pinene (18.1%)	GC and GC-MS	[32]
Sepal	Jordan	Irano-Turanian	Full maturation period	EO	*trans*-Sabinene hydrate (58.8%), terpinolene (5.0%), *E*-*β*-ocimene (4.1%), p-methyl-acetophenone (3.2%), germacrene D (3.1%), *Z*-*β*-ocimene (4.9%), *δ*-selinene (2.0%), *γ*-terpinene (1.7%), *δ*-cadinene (1.3%), *E*-caryophyllene (5.6%)	GC and GC-MS	[32]
Aerial parts	Algeria	Mogheul	April 2011	EO	Germacrene D (20.5%), *β*-caryophyllene (3.8%), beta-cubebene (2.7%), *δ*-cadinene (2.6%), 1,10-di-epi-cubenol (2. 6%), *γ*-cadinene (2.5%), (E)-*β*-farnesene (3.5%), bicyclogermacrene (2.2%), *α*-muurolol (2.1%), *α*-copaene (10.4%), *β*-phellandrene (3.8%)	GC and GC-MS	[36]
Seeds	Spain	—	—	EO	Camphor (38.94%), 13-*epi*-manool (5.61%), 𝛿-elemene (3.93%), beta-eudesmol (3.76%), *n*-undecane (2.65%), *α*-terpinyl acetate (4.77%), linalyl acetate (2.53%), neryl acetate (2.40%), *α*-terpineol (2.03%), caryophyllene oxide (7.28%)	GC-MS and GC-FID	[33]
Aerial parts	Greece	Crete Island	Blossoming (April 2004)	EO	Beta-phellandrene (30.3%), methyl ester of 6-octadecenoic acid (15.0%), camphor (7.0%), (*Z*)-*β*-ocimene (6.6%), fenchone (9.4%), isopropyl ester (7.8%), aromadendrene (4.0%), *α*-humulene (3.7%), (*E*)-caryophyllene (16.1%)	GC and GC-MS	[34]
Aerial parts (fresh)	Sicily	Piano Battaglia	Full flowering stage (July 2009)	EO	Hexadecanoic acid (23.1%), ethyl hexadecanoate (2.6%), benzaldehyde (7.3%), 9,12,15-octadecatrienal (2.9%), limonene (2.0%), (*E*)-*β*-ionone (1.9%), (*Z*)-9-octadecenoic acid (11.9), phenyl acetaldehyde (1.5%), (*E*)-caryophyllene (1.2%), *β*-phellandrene (5.9%)	GC and GC-MS	[8]
Aerial parts	Algeria	Djelfa	March 2019	EO	*cis*-Muurola-3,5-diene (14.6%), unknown (10.5%), bicyclogermacrene (6.8%), bicycloelemene (4.3%), *γ*-cadinene (4.8%), *β*-pinene (4.2%), 2,3-dehydro-1,4-cineol (3.7%), *α*-cubebene (3.0%), *α*-pinene (2.8%), *γ*-amorphene (10.5%)	GC and GC-MS	[35]
Leaves and flowers (dried)	Turkey	Kütahya-Gediz	2016-2017	EO	Linalyl acetate (81.97%), *β*-myrcene (2.73%), *n*-pentanal (0.42%), beta-ocimene (0.39%), hexanal (0.34%), *α*-pinene (0.34%), limonene (1.14%), *trans*-caryophyllene (0.32%), *β*-pinene (0.31%), linalool (8.66%)	GC and GC-MS	[37]
Aerial parts (wild)	Sicily	Piano Battaglia	Full flowering stage (July 2009)	EO	Hexadecanoic acid (23.1%), benzaldehyde (7.3%), b-phellandrene (5.9%), limonene (2.0%), 9,12,15-octadecatrienal (2.9%), ethyl hexadecanoate (2.6%), caryophyllene oxide (1.9%), (*E*)-*b*-ionone (1.9%), spathulenol (1.7%), (*Z*)-9-octadecenoic acid (11.1%)	GC and GC-MS	[19]
Aerial parts (cultivated)	Sicily	Piano Battaglia	July 2010	EO	Hexadecanoic acid (11.0%), (*E*)-*b*-ionone (3.9%), (*Z*)-9-octadecenoic acid (5.6%), *b*-phellandrene (4.1%), caryophyllene oxide (2.8%), (*E*)-caryophyllene (3.8%), methyl hexadecanoate (3.8%), carvacrol (2.4%), spathulenol (2.0%), hexahydrofarnesyl acetone (9.7%)	GC and GC-SM	[19]
Fruits	Tunisia	Sabelet Ben Ammar	Full fruit ripening stage	EO	*β*-Caryophyllene (23.1%), camphene (6.5%), *α*-humulene (5.6%), germacrene D (3.5%), viridiflorol (4.3%), 1-octen-3-ol (3.9%), (*E*)-*β*-ocimene (1.5%), 1,8-cineole (3.0%), manool (1.1%), caryophyllene oxide (15.9%)	GC and GC-MS	[33]
Stems	Tunisia	Sabelet Ben Ammar	Full fruit ripening stage		Camphor (10.9%), terpinolene (6.6%), methyl eugenol (6.1%), *α*-pinene (5.9%), *α*-thujone (3.1%), 1,8-cineole (5.8%), caryophyllene oxide (4.5%), aromadendrene (3.6%), epi-13-manool (2.3%), viridiflorol (10.3%)	GC and GC-MS	[33]
Leaves	Tunisia	Sabelet Ben Ammar	Full fruit ripening stage		epi-13-Manool (13.7%), camphor (3.9%), caryophyllene oxide (3.9%), *α*-pinene (3.4%), p-cymen-8-ol (3.7%), terpinen-4-ol (3.6%), 1,8-cineole (3.0%), eugenol (2.8%), (*E*)-*β*-ocimene (2.6%), manool (11.0%)	GC and GC-MS	[33]
Aerial parts	Tunisia	Sabelet Ben Ammar	Full fruiting stage (April 2007)	EO	Viridiflorol (21.6%), methyl eugenol (9.4%), *α*-terpineol (5.3%), spathulenol (3.7%), *β*-caryophyllene (7.1%), caryophyllene oxide (2.4%), epi-13-manool (2.2%), germacrene D (1.9%), eugenol (1.8%), camphene (17.6%)	GC and GC-MS	[33]
Aerial parts	Tunisia	Sers	Full fruiting stage (April 2007)		(*Z*)-*β*-ocimene (29.5%), beta-thujone (7.9%), *α*-pinene (5.5%), tricyclene (5.1%), 18-cineole (1.9%), *α*-calacorene (2.5%), terpinen-4-ol (2.1%), germacrene D (3.1%), *β*-caryophyllene (1.8%), *β*-phellandrene (8.2%)	GC and GC-MS	[33]
Aerial parts	Tunisia	Somaa			Tricyclene (18.8%), nonane (10.3%), terpinolene (7.3%), -terpineol (2.2%), bornyl acetate (4.9%), camphor (2.9%), *α*-terpinyl acetate (3.5%), limonene (2.3%), *α β*-eudesmol (2.2%), methyl eugenol (7.7%)	GC and GC-MS	[33]
Seeds	Tunisia	Sabelet Ben Ammar	Full ripeness (April 2007)	EO	Camphor (33.83%), caryophyllene oxide (10.11%), octane (4.78%), 13-epi-manool (3.57%), hexanal (2.46%), *β*-bisabolene (1.84%), *α*-terpineol (3.24%), tricyclene (5.54%), *α*-copaene (3.19%), *α*-thujene (13.36%)	GC-MS and GC-FID	[33]
Seeds	Tunisia	Sabelet Ben Ammar	Full ripeness (April 2007)	Lipid extraction	Palmitic acid (9.25%), stearic acid (2.48%), linolenic acid (45.89%), arachidic acid (0.20%), C18:3n-3/C18:2n-6 (1.67%), SFA (11.93%), USFA (88.07%), oleic acid (14.67%), linoleic acid (27.39%), palmitoleic acid (0.12%)	GC and GC-MS	[33]
Seeds	Tunisia	Sers	Full ripeness (April 2007)	EO	*β*-Pinene (48.08%), epi-cubebol (10.74%), *β*-eudesmol (1.00%), *α*-bisabolol (2.97%), caryophyllene oxide (2.90%), spathulenol (0.93%), eugenol (0.97%), geraniol (0.95%), borneol (1.97%), germacrene D (2.09%)	GC and GC-MS	[33]
Seeds	Tunisia	Sers	Full ripeness (April 2007)	Lipid extraction	Palmitic acid (9.63%), oleic acid (14.14%), linoleic acid (23.79%), linolenic acid (42.84%), SFA (18.35%), USFA (81.65%), stearic acid (4.22%), arachidic acid (4.50%), C18:3n-3/C18:2n-6 (1.53%), palmitoleic acid (0.89%)	GC and GC-MS	[33]
Seeds	Tunisia	Somaa	Full ripeness (April 2007)	EO	Octane (27.39%), *δ*-cadinene (5.77%), p-cymene (1.64%), camphor (3.53%), bicyclogermacrene (1.86%), *β*-pinene (3.74%), *α*-terpineol (1.38%), limonene (0.79%) n-nonane (18.01%), epi-cubebol (9.02%)	GC and GC-MS	[33]
Seeds	Tunisia	Somaa	Full ripeness (April 2007)	Lipid extraction	Palmitic acid (12.11%), stearic acid (3.02%), linoleic acid (25.33%), arachidic acid (1.30%), SFA (16.43%), linolenic acid (41.71%), oleic acid (15.51%), USFA (83.57%), C18:3n-3/C18:2n-6 (1.65%), palmitoleic acid (1.02%)	GC and GC-MS	[33]
Aerial part	Algeria	Bordj Bou Arreridj	Flowering stage (spring April-May)	Crude extract (CrE)	Flavonoids (08.40 ± 0.32 mg EQ/g E), polyphenols (177.56 ± 2.51 mg EGA/g E)	Spectrophotometrically	[21]
Aerial part	Algeria	Bordj Bou Arreridj		Chloroform extract (ChE)	Flavonoids (14.87 ± 0.81 mg EQ/g E), polyphenols (156.81 ± 1.57 mg EGA/g E)	Spectrophotometrically	[21]
Aerial part	Algeria	Bordj Bou Arreridj		Ethyl acetate extract (EAE)	Flavonoids (28.81 ± 0.38 mg EQ/g E), polyphenols (661.78 ± 4.00 mg EGA/g E)	Spectrophotometrically	[21]
Aerial part	Algeria	Bordj Bou Arreridj		Aqueous extract (AqE)	Flavonoids (06.74 ± 0.14 mg EQ/g E), polyphenols (123.18 ± 4.20 mg EGA/g E)	Spectrophotometrically	[21]
Aerial part	Algeria	Laghouat	May 2004	80% (*v*/*v*) aqueous methanol	Flavonoids (3.04 ± 0.01 mg RE/g dw), total phenols (7.2 ± 0.04 mg GAE/g dw), flavonols (0.85 ± 0.001 mg QE/g dw)	Spectrophotometrically	[12]
Aerial part	Algeria	Setif and Batna	2016	Decoction	Total phenols (129.02 ± 2.67 mg GAE/g DW), total flavonoid contents (18.62 ± 0.06 mg QE/g DW), total tannin contents (73.80 ± 2.23 mg TAE/g DW) Total carotenoid contents (0.92 ± 0.041 mg/g DW) Total chlorophyll A (1.21 ± 0.02 mg/g DW) Total chlorophyll B (2.48 ± 0.04 mg/g DW)	Spectrophotometrically	[13]
Aerial part	Algeria	Setif and Batna	2016	Methanol extract (85%)	Total phenols (190.16 ± 1.74 mg GAE/g DW) Total flavonoid contents (23.50 ± 0.71 mg QE/g DW) Total tannin contents (118.88 ± 1.25 mg TAE/g DW) Total carotenoid contents (0.58 ± 0.005 mg/g DW) Total chlorophyll A (1.67 ± 0.02 mg/g DW) Total chlorophyll B (0.63 ± 0.01 mg/g DW)	Spectrophotometrically	[13]
Aerial part	Turkey	Artvin	06th September 2004	Methanol extracts	Rosmarinic acids (29.30 ± 0.24 *μ*g mg^_1^)	Spectrophotometrically	[38]
					Rosmarinic acids (26.12 ± 0.73 *μ*g mg^_1^)	HPLC	[6]
Aerial parts	Tunisia	Tunis (higher semiarid)	Flowering stage (March and April 2008)	Methanolic extracts	*Phenolic acids* p-Hydroxybenzoïc acids (229.87 ± 8.60 *μ*g/g), p-coumaric acid (77.65 ± 5.67 *μ*g/g), rosmarinic acid (1688.01 ± 63.42 *μ*g/g), vanillic acid (20.21 ± 0.46 *μ*g/g), caffeic acids (97.29 ± 2.86 *μ*g/g), ferulic acids (40.41 ± 3.32 *μ*g/g) *Phenolic diterpenes* Carnosic acids (63.52 ± 15.30 *μ*g/g), methyl carnosate contents (633.37 ± 11.66 *μ*g/g), carnosol (25.52 ± 7.27 *μ*g/g) *Flavonoids* Naringenins (940.41 ± 22.50 *μ*g/g), cirsiliols (73.16 ± 1.72 *μ*g/g), luteolins (13.84 ± 2.62 *μ*g/g), apigenins (3.01 ± 0.69 *μ*g/g), naringins (57.30 ± 3.55 *μ*g/g), hesperidins (21.74 ± 3.2 *μ*g/g), genkwanins (2.80 ± 0.72 *μ*g/g)	HPLC-UV	[6]
Aerial parts	Tunisia	Bir Mroua (subhumid)	Flowering stage (March and April 2008)	Methanolic extracts	*Phenolic acids* p-Hydroxybenzoïc acids (382.79 ± 11.98 *μ*g/g), caffeic acid (191.19 ± 27.72 *μ*g/g), rosmarinic acid (2503.96 ± 224.40 *μ*g/g), p-coumaric acid (133.78 ± 1.88 *μ*g/g), ferulic acid (72.89 ± 0.86 *μ*g/g), vanillic acid (14.51 ± 0.46 *μ*g/g) *Phenolic diterpenes* Carnosic acids (67.95 ± 3.73 *μ*g/g), carnosols (32.09 ± 1.46 *μ*g/g) *Flavonoids* Naringenins (1402.07 ± 5.17 *μ*g/g), luteolins (21.14 ± 2.03 *μ*g/g), hesperidins (84.48 ± 4.67 *μ*g/g), apigenins (13.56 ± 0.51 *μ*g/g), cirsiliols (53.18 ± 3.15 *μ*g/g), genkwanins (2.53 ± 0.57 *μ*g/g), naringins (36.79 ± 2.83 *μ*g/g)	HPLC-UV	[6]
Aerial parts	Tunisia	Hencha (higher arid)	Flowering stage (March and April 2008)	Methanolic extracts	*Phenolic acids* p-Hydroxybenzoic acids (51.18 ± 3.76 *μ*g/g), caffeic acids (50.77 ± 3.04 *μ*g/g), ferulic acids (74.55 ± 16.66 *μ*g/g), p-coumaric acids (22.51 ± 0.84 *μ*g/g), rosmarinic acids (475.74 ± 7.45 *μ*g/g), vanillic acids (9.59 ± 0.91 *μ*g/g) *Phenolic diterpenes* Methyl carnosate (1159.73 ± 41.68 *μ*g/g), carnosic acids (55.47 ± 1.60 *μ*g/g) *Flavonoids* Naringenins (254.82 ± 22.14 *μ*g/g), cirsiliols (57.89 ± 3.81 *μ*g/g), luteolins (51.65 ± 2.42 *μ*g/g), apigenins (23.95 ± 1.00 *μ*g/g), genkwanins (2.65 ± 0.12 *μ*g/g), hesperidins (24.19 ± 1.21 *μ*g/g), naringins (20.26 ± 0.50 *μ*g/g)	HPLC	[6]
Aerial parts (dried)	Saudi Arabia	Assir	18th February 2001	Alcoholic extract	Verbenacines and salvinines	1D and 2D NMR	[39]
Roots (dried)	Algeria	Batna	—	Acetone extract	6,7-Dehydroroyleanones, cryptanol, sitosterols, campesterols, 6-hydroxysalvonolones, microstegiols, stigmasterols	IR, UV, 1H 13C NMR, and NMR	[40]

**Table 3:** Antibacterial potential of *S. verbenaca* extracts and EOs.

Plant section	Extracts	Methodology	Tested bacterial strains	Antibacterial results	Ref.
Aerial parts	Ethanolic extract	Disc diffusion method dose (20 *μ*L)	Gram positive *Staphylococcus aureus* (ATCC 25923) *Micrococcus luteus* (NRRL B-4375) *Staphylococcus aureus* (MU 44) *Staphylococcus aureus* (MU 38) *Staphylococcus epidermidis* (MU 30) *Bacillus subtilis* (ATCC 6633) *Streptococcus mutans* (CNCTC 8/77) Gram negative *Escherichia coli* (ATCC 25922) *Pseudomonas aeruginosa* (ATCC 27853) *Stenotrophomonas maltophilia* (MU 99) *Chryseomonas luteola* (MU65) *Pseudomonas fluorescens* (MU 87) *Stenotrophomonas maltophilia* (MU 64) *Pseudomonas stutzeri* (MU 70)	*Ф* = 11 mm No inhibition *Ф* = 10 mm *Ф* = 9 mm *Ф* = 9 mm *Ф* = 9 mm No inhibition No inhibition No inhibition No inhibition No inhibition No inhibition No inhibition No inhibition	[10]
Not specified	Methanolic extract (80%) Ethanolic extract (80%)	Not specified	Not specified	The 80% methanol extract prepared using ultrasound extraction showed the highest antimicrobial activity	[41]
Aerial parts	Methanolic extract	Minimum inhibitory concentration	Gram positive *Micrococcus sedentarius* (L7B5) *Staphylococcus xylosus* (IP8166) *Corynebacterium* gr. C (L3C3) *Staphylococcus cohnii* (L6S3) *Corynebacterium* gr. D2 (L19C1) *Micrococcus luteus* (L1C5) *Corynebacterium xerosis* (IP5216) *Staphylococcus epidermidis* (L1S2) *Staphylococcus intermedius* (IP8160) *Corynebacterium* gr. B (L16C3) Gram negative *Acinetobacter* sp. (LH5DC1)	MIC = 500 *μ*g/mL MIC > 1000 *μ*g/mL MIC = 500 *μ*g/mL MIC = 500 *μ*g/mL MIC = 500 *μ*g/mL MIC > 1000 *μ*g/mL MIC = 500 *μ*g/mL MIC = 500 *μ*g/mL MIC > 1000 *μ*g/mL MIC > 1000 *μ*g/mL	[42]
			*Moraxella* sp. (LH7SV1) *Alcaligenes* sp. (LH4TV1) *Pseudomonas cepacia* (V6108) *Pseudomonas aeruginosa* (V5791)	MIC = 700 *μ*g/mL MIC > 1000 *μ*g/mL MIC > 1000 *μ*g/mL MIC > 1000 *μ*g/mL MIC > 1000 *μ*g/mL	
Aerial parts	Methanol : chloroform (1 : 1, *v*/*v*) extract	Microdilution assay	Gram positive *Bacillus cereus* (ATCC 11778) *Staphylococcus aureus* (ATCC 25923) Gram negative *Klebsiella pneumoniae* (NTCC 9633) *Escherichia coli* (ATCC 8739)	MIC = 2.0 mg/mL MIC = 3.0 mg/mL MIC = 2.0 mg/mL MIC = 8.0 mg/mL	[17]
Aerial parts	Methanolic extract subfractions: Crude extract (CrE) Chloroform extract (ChE) Ethyl acetate extract (EAE) Aqueous extract (AqE)	Disc diffusion method Dose (3 mg and 6 mg/disc)	Gram positive *Staphylococcus aureus* (ATCC 52952)	EAE *Ф* (3 mg/disc) = 12 mm *Ф* (6 mg/disc) = 16 mm ChE *Ф* (3 mg/disc) = 11 mm *Ф* (6 mg/disc) = 10 mm CrE $\underset{¯}{Ф}\;\left(3\text{ mg or }6\text{ mg}/\text{disc}\right)=11\text{ mm}$ AqE: no inhibition	[21]
			*Bacillus cereus* (ATCC 10876)	EAE *Ф* (3 mg/disc) = 13 mm *Ф* (6 mg/disc) = 15 mm ChE *Ф* (3 mg/disc) = 11 mm *Ф* (6 mg/disc) = 15 mm CrE *Ф* (3 mg/disc) = no inhibition *Ф* (6 mg/disc) = 12 mm AqE: no inhibition	
			*Enterococcus faecalis* (ATCC 49452)	EAE *Ф* (3 mg/disc) = 12 mm *Ф* (6 mg/disc) = 14 mm ChE *Ф* (3 mg/disc) = 09 mm *Ф* (6 mg/disc) = 12 mm CrE *Ф* (3 mg/disc) = no inhibition *Ф* (6 mg/disc) = 11 mm AqE: no inhibition	
			*Listeria monocytogenes* (ATCC 15313)	EAE *Ф* (3 mg/disc) = 10 mm *Ф* (6 mg/disc) = 14 mm ChE *Ф* (3 mg/disc) = 8.0 mm *Ф* (6 mg/disc) = no inhibition CrE *Ф* (3 mg/disc) = no inhibition *Ф* (6 mg/disc) = 12 mm AqE: no inhibition	
			Gram negative *Escherichia coli* (ATCC 25922)	EAE *Ф* (3 mg/disc) = 11 mm *Ф* (6 mg/disc) = 14 mm ChE *Ф* (3 mg/disc) = 09 mm *Ф* (6 mg/disc) = 12 mm CrE and AqE No inhibition	
			*Pseudomonas aeruginosa* (ATCC 27853)	EAE *Ф* (3 mg/disc) = 12 mm *Ф* (6 mg/disc) = 15 mm ChE *Ф* (3 mg/disc) = no inhibition *Ф* (6 mg/disc) = 13 mm CrE *Ф* (3 mg/disc) = no inhibition *Ф* (6 mg/disc) = 9 mm AqE: no inhibition	
			*Citrobacter freundii* (ATCC 8090)	EAE *Ф* (3 mg/disc) = 12 mm *Ф* (6 mg/disc) = 14 mm ChE *Ф* (3 mg/disc) = no inhibition *Ф* (6 mg/disc) = 14 mm CrE *Ф* (3 mg/disc) = 11 mm *Ф* (6 mg/disc) = no inhibition AqE: no inhibition	
			*Acinetobacter baumannii* (ATCC 19306)	EAE *Ф* (3 mg/disc) = 10 mm *Ф* (6 mg/disc) = 15 mm ChE *Ф* (3 mg/disc) = no inhibition *Ф* (6 mg/disc) = 14 mm CrE *Ф* (3 mg/disc) = no inhibition *Ф* (6 mg/disc) = 10 mm AqE: no inhibition	
			*Proteus mirabilis* (ATCC 35659)	EAE *Ф* (3 mg or 6 mg/disc) = 13 mm ChE *Ф* (3 mg/disc) = no inhibition *Ф* (6 mg/disc) = 13 mm CrE and AqE No inhibition	
			*Salmonella typhi* (ATCC 13311)	No inhibition	
Leaves	Ethyl acetate extract	Agar diffusion test Dose (100 *μ*g and 300 *μ*g/disc) Microbroth dilution assay	Gram positive *Bacillus brevis* (ATCC 9999) *Bacillus subtilis* (ATCC 6633) *Staphylococcus aureus* (ATCC 43300) Gram negative *Klebsiella pneumoniae* (ATCC13883) *Escherichia coli* (ATCC 25922)	MIC = 50 *μ*g/mL MIC = 50 *μ*g/mL No inhibition No inhibition No inhibition	[7]
Aerial parts	Essential oil	Broth dilution method	Gram positive *Bacillus subtilis* (ATCC6633) *Staphylococcus aureus* (ATCC 25923) *Staphylococcus epidermidis* (ATCC 12228) *Streptococcus faecalis* (ATTC 29212)	MIC = 50 *μ*g/mL MIC = 100 *μ*g/mL MIC = 50 *μ*g/mL MIC = 100 *μ*g/mL	[8]
			Gram negative *Escherichia coli* (ATCC25922) *Proteus vulgaris* (ATCC13315) *Klebsiella pneumoniae* (ATCC10031) *Pseudomonas aeruginosa* (ATCC27853)	MIC > 100 *μ*g/mL MIC > 100 *μ*g/mL MIC > 100 *μ*g/mL MIC > 100 *μ*g/mL	

*Ф*: diameter of inhibition.

**Table 4:** Antioxidant activity of *S. verbenaca.*

Part used	Extracts	Methods used	Key results	Ref.
Not specified	Methanolic extract (80%) Ethanolic extract (80%)	DPPH assay *β*-Carotene/linoleic acids	The 80% methanol extract prepared by maceration was highly active The 80% of ethanol extract was the most active	[41]
Aerial parts (stems and leaves)	Hydromethanolic extract	Oxygen consumption	A strong inhibition of oxygen consumption (92%)	[44]
		Conjugated diene formation (CD)	A strong inhibition of CD formation of LDL peroxidation (92%)	
		Thiobarbituric acid reactive substance (TBARS) formation	A strong inhibition of TBARS formation of linolenic acid oxidation (93%)	
Not specified	Methanolic extract	DPPH assay *β*-Carotene–linoleic acid method	IC_50_ = 14.30 ± 1.42 *μ*g/mg Percent inhibition = 77.03 ± 0.42%	[38]
Aerial parts	Methanolic extract	DPPH assay	IC_50_ = 86.9 *μ*g/mL	[42]
		ABTS assay	IC_50_ at 5 min = 777.3 *μ*g/mL TEAC at 5 min = 0.624 IC_50_ at 20 min = 499.5 *μ*g/mL TEAC at 10 min = 0.647 TEAC at 20 min = 0.705 TEAC at 15 min = 0.705	
Aerial parts	Methanolic extract from postdistilled plant	DPPH method	Sers: IC_50_ = 24.47 ± 1.87 *μ*g/mL Touiref: IC_50_ = 25.11 ± 2.97 *μ*g/mL Beja: IC_50_ = 26.62 ± 0.8 *μ*g/mL Chott Meriem: IC_50_ = 28.28 ± 0.16 *μ*g/mL Tunis: IC_50_ = 30.34 ± 2.28 *μ*g/mL Rass Zebib: IC_50_ = 31.19 ± 2.25 *μ*g/mL Bou Arada: IC_50_ = 33.47 ± 4.13 *μ*g/mL Bir Mroua: IC_50_ = 34.70 ± 2.43 *μ*g/mL Hencha: IC_50_ = 39.85 ± 3.9 *μ*g/mL Enfidha: IC_50_ = 40.91 ± 0.5 *μ*g/mL	[6]
		ABTS method	Hencha: TEAC = 120.11 ± 6.62 *μ*M trolox/mg Enfidha: TEAC = 134.45 ± 5.27 *μ*M trolox/mg Bir Mroua: TEAC = 139.26 ± 10.59 *μ*M trolox/mg Rass Zebib: TEAC = 144.02 ± 3.4 *μ*M trolox/mg Bou Arada: TEAC = 154.97 ± 6.79 *μ*M trolox/mg Tunis: TEAC = 190.51 ± 6.71 *μ*M trolox/mg Chott Meriem: TEAC = 196.72 ± 1.61 *μ*M trolox/mg Sers: TEAC = 271.51 ± 4.52 *μ*M trolox/mg Beja: TEAC = 282.17 ± 6.58 *μ*M trolox/mg Touiref: TEAC = 287.81 ± 3.65 *μ*M trolox/mg	
		FRAP	Beja: 142.07 ± 1.46 mM Fe^+2^/mg Sers: 139.09 ± 11.23 mM Fe^+2^/mg Touiref: 131.86 ± 1.05 mM Fe^+2^/mg Chott Meriem: 124.27 ± 0.38 mM Fe^+2^/mg Tunis: 122.33 ± 3.7 mM Fe^+2^/mg Bou Arada: 120.53 ± 7.53 mM Fe^+2^/mg Rass Zebib: 118.02 ± 15.25 mM Fe^+2^/mg Bir Mroua: 109.22 ± 5.04 mM Fe^+2^/mg Hencha: 104.89 ± 0.37 mM Fe^+2^/mg Enfidha: 101.46 ± 1.97 mM Fe^+2^/mg	
Aerial parts	Crude extract	DPPH method	IC_50_ = 47.50 *μ*g/mL	[14]
Aerial parts	Methanolic extract	DPPH FRAP	IC_50_ = 9.79 ± 0.47 *μ*g/mL High reducing power	[43]
Not specified	Methanolic extract	DPPH method	IC_50_ = 16.92 ± 0.2 *μ*M	[12]
Aerial parts	Methanolic extract subfractions: Crude extract (CrE) Chloroform extract (ChE) Ethyl acetate extract (EAE) Aqueous extract (AqE)	DPPH method	EAE: IC_50_ = 0.0086 mg/mL CrE: IC_50_ = 0.0336 mg/mL ChE: IC_50_ = 0.0725 mg/mL AqE: IC_50_ = 0.0389 mg/mL	[21]
		Reducing power method	EAE: EC_50_: 0.0047 mg/mL CrE: EC_50_: 0.0453 ± 0.000 mg/mL AqE: EC_50_: 0.0455 mg/mL	
		Metal chelating method	AqE and CrE reported the highest activity EAE chelation did not exceed 20%	
Aerial parts	Methanolic extracts (85%) (ME) Decoction extract (distilled water) (DE)	DPPH method	ME: IC_50_: 24.36 ± 1.13 *μ*g/mL DE: IC_50_: 27.26 ± 1.05 *μ*g/mL	[13]
		ABTS method	ME: IC_50_: 19.96 ± 1.03 *μ*g/mL DE: IC_50_: 36.86 ± 1.03 *μ*g/mL	
		Alkaline DMSO superoxide radical scavenging	ME: IC_50_: 07.77 ± 1.00 *μ*g/mL DE: IC_50_: 18.78 ± 1.07 *μ*g/mL	
		*β*-Carotene bleaching	DE: inhibition: 96.12 ± 2.48% ME: inhibition: 82.58 ± 2.39%	
		Reducing power method	DE: EC_50_: 69.52 ± 3.07 *μ*g/mL ME: EC_50_: 56.64 ± 4.81 *μ*g/mL	
		Metal chelating activity method	ME: IC_50_: 70.39 ± 1.13 *μ*g/mL DE: IC_50_: 109.70 ± 1.72 *μ*g/mL	
		Phenanthroline method	ME: IC_50_: 27.03 ± 1.54 *μ*g/mL DE: IC_50_: 40.26 ± 0.59 *μ*g/mL	
		Cupric reducing antioxidant capacity (CUPRAC)	ME: A_0.50_: 14.66 ± 2.51 *μ*g/mL DE: A_0.50_: 33.00 ± 0.30 *μ*g/mL	
Root	Methanolic extract	H2DCF-DA method	Significant reduction in the intracellular reactive oxygen species (ROS) level for both tested values (1 and 10 *μ*g/mL)	[14]

**Table 5:** Anticancer effects of *S. verbenaca*.

Plant part	Tested extract	Cell lines	Major results	Ref.
Leaves	Ethyl acetate	Human breast adenocarcinoma	IC_50_: 41.3 ± 4.8 *μ*g/mL	[7]
Aerial parts	Methanol	Human colon adenocarcinoma	LC_50_: 60.4 *μ*g/mL	[15]
		Human hepatoblastoma	LC_50_: 68.9 *μ*g/mL	
		Human breast cancer cells	LC_50_: 43.1 *μ*g/mL	
		Human pancreatic carcinoma	LC_50_: 42.2 *μ*g/mL	
Aerial parts	Hexane	Human embryonal rhabdomyosarcoma cancerous cell lines	IC_50_: 474.6 ± 1.3 *μ*g/mL	[16]
		Vero (monkey kidney cancerous cell lines)	IC_50_ > 500 *μ*g/mL	
Aerial parts	Ethyl acetate	Human embryonal rhabdomyosarcoma cancerous cell lines	IC_50_ > 500 *μ*g/mL	[16]
		Vero (monkey kidney cancerous cell lines)	IC_50_: 223.6 ± 1.6 *μ*g/mL	
Aerial parts	*n*-Butanol	Human embryonal rhabdomyosarcoma cancerous cell lines	IC_50_ > 500 *μ*g/mL	[16]
		Vero (monkey kidney cancerous cell lines)	IC_50_ > 500 *μ*g/mL	
Aerial parts	Methanol and chloroform	Breast adenocarcinoma	IC_50_: 31.5 ± 13.7 *μ*g/mL	[17]
		Colon adenocarcinoma	IC_50_: 50.0 ± 5.3 *μ*g/mL	
		Glioblastoma	IC_50_ was not calculated	
		Human kidney epithelial cell line	IC_50_: 20.8 ± 2.5 *μ*g/mL	
Leaves	Methanol	Monkey kidney cells	CC_50_: 64 *μ*g/mL	[18]
		Human larynx cancer cells	CC_50_ = 64 *μ*g/mL	
Roots	Methanol	Human monocytic leukemia cell line	70% of apoptosis and 30% of viable cells at a 1000 *μ*g/mL concentration	[23]
Aerial parts	Essential oils	Human melanoma cell line	IC_50_ = 8.1 ± 0.6 *μ*g/mL	[19]

**Table 6:** Antiparasitic activity of *S. verbenaca*.

Activity	Part used	Extract	Parasite	Major results	Ref.
Antileishmanial activity	Whole plant part	*n-*Hexane	*Leishmania major*	IC_50_: 155.4 *μ*g/mL	[20]
			*Leishmania tropica*	IC_50_: 148.2 *μ*g/mL	
			*Leishmania infantum*	IC_50_: 14.1 *μ*g/mL	
		Dichloromethane	*Leishmania major*	IC_50_: 24.5 *μ*g/mL	
			*Leishmania tropica*	IC_50_: 33.7 *μ*g/mL	
			*Leishmania infantum*	IC_50_: 31.5 *μ*g/mL	
		Methanol	*Leishmania major*	IC_50_ > 1000 *μ*g/mL	
			*Leishmania tropica*	IC_50_: 850.7 *μ*g/mL	
			*Leishmania infantum*	IC_50_ > 1000 *μ*g/mL	
Antimalarial activity	Aerial parts	Methanol chloroform	*Plasmodium falciparum* (FCR-3 strain)	IC_50_: 23.9 ± 1.1 *μ*g/mL	[11]

**Table 7:** Other biological activities of *S. verbenaca*.

Activity	Part used	Extracts	Experiment	Major results	Ref.
Antihemolytic	Aerial part	Ethyl acetate	2,2-Azobis (2-amidinopropane) dihydrochloride induces erythrocyte oxidative hemolysis (AAPH)	HT50: 165 min	[21]
		Crude		HT50: 125.1 min	
		Chloroform		HT50: 111.5 min	
		Aqueous		HT50: 111.5 min	
Xanthine oxidase inhibition	Aerial part	Chloroform	Colorimetric approach based on uric acid generation at 295 nm in the presence of 100 mM xanthine in phosphate buffer	IC_50_: 0.0088 ± 0.0 mg/mL	
		Ethyl acetate		IC_50_: 0.0165 ± 0.001 mg/mL	
		Crude		IC_50_: 0.0520 ± 0.003 mg/mL	
		Aqueous		IC_50_: 0.9800 ± 0.004 mg/mL	
Porcine liver carboxylesterase inhibition	Aerial part	Aqueous methanol	Enzyme inhibition by spectrophotometric assay	CE (carboxylesterase) inactivation with a pI = 5.1 and a Ki value of 38 Mm	[12]
Healing of burns	Leaves	Hexane	Second-degree burn injury induced by a hot metal cylinder in rats	Accelerated healing process with 44.34%	[16]
		Ethyl acetate		Accelerated healing process with 47.55%	
		*n*-Butanol		Accelerated healing process with 49.16%	
Anticholinesterases	Aerial part	Methanol	Cholinesterase inhibition	Inhibition effect of AChE at 100 *μ*g/mL	[13]
Anti-*α*-amylase			*α*-Amylase inhibition	IC_50_: 01.3 ± 0.08 *μ*g/mL	
Anti-*α*-glucosidase			*α*-Glucosidase inhibition	IC_50_ = 150.5 ± 1.4 *μ*g/mL	
Immunomodulatory	Aerial parts	Methanol	Phagocytic activity used carbon clearance rate test	Significantly increased phagocytic index (0.095 ± 0.012) at a dose of 200 mg/kg Increased corrected phagocytic index *α* (0.095 ± 1.71)	[14]

**Table 8:** Toxicological studies of *S. verbenaca*.

Activities	Part used	Extract	Experimental approach	Major results	Ref.
Acute oral toxicity	Aerial parts	*n*-Butanol, hexane, ethyl acetate	Orally delivered at a dose of 2000 mg/kg in a volume of 0.25 mL per 20 g of body weight to mice and examined for 14 days	LD_50_ > 2000 mg/kg body weight	[64]
Acute dermal toxicity	Aerial parts	Hexane, ethyl acetate, *n*-butanol	For 14 days, daily topical application of *S. verbenaca* extracts at a dose of 2000 mg/kg body weight	There are no adverse effects, behavioral problems, or fatalities	[64]
Subchronic dermal toxicity	Aerial parts	Hexane, ethyl acetate, *n*-butanol	For 28 days, daily topical application of *S. verbenaca* extracts at a dose of 2000 mg/kg body weight	There are no harmful symptoms or changes in the amount of water or food consumed There is no lethality There is no change in the parameters of fasting blood circulation There were no morphological alterations in the main vital organs investigated	[64]

## Data Availability

All the data are cited in the main text of this document.
